The article "Panax ginseng C. A. Meyer Phenolic Acid Extract Alleviates Ultraviolet B-Irradiation-Induced Photoaging in a Hairless Mouse Skin Photodamage Model" was published in 2021. Journal: Evid Based Complement Alternat Med.

# *Panax ginseng* C. A. Meyer Phenolic Acid Extract Alleviates Ultraviolet B-Irradiation-Induced Photoaging in a Hairless Mouse Skin Photodamage Model

**DOI:** 10.1155/2021/9962007

**Published:** 2021-08-02

**Authors:** Zhenzhuo Li, Rui Jiang, Jianzeng Liu, Xiaohao Xu, Liwei Sun, Daqing Zhao

**Affiliations:** ^1^Jilin Ginseng Academy, Changchun University of Chinese Medicine, Changchun, Jilin 130117, China; ^2^Research Center of Traditional Chinese Medicine, The Affiliated Hospital to Changchun University of Chinese Medicine, Changchun, Jilin 130021, China; ^3^Key Laboratory of Active Substances and Biological Mechanisms of Ginseng Efficacy, Ministry of Education, Changchun University of Chinese Medicine, Changchun, Jilin 130117, China; ^4^Jilin Province Traditional Chinese Medicine Characteristic Health Product Research and Development Cross-Regional Cooperation Science and Technology Innovation Center, Changchun University of Chinese Medicine, Changchun, Jilin 130117, China

## Abstract

Here, we evaluated the *in vivo* skin-protective effects of topical applications of *Panax ginseng* C. A. Meyer extract (PG2) and its phenolic acid- (PA-) based components against UVB-induced skin photoaging. PG2 or PA applied to skin of hairless mice after UVB-irradiation alleviated UVB-induced effects observed in untreated skin, such as increased transepidermal water loss (TEWL), increased epidermal thickness, and decreased stratum corneum water content without affecting body weight. Moreover, PG2 and PA treatments countered reduced mRNA-level expression of genes encoding filaggrin (FLG), transglutaminase-1 (TGM1), and hyaluronan synthases (HAS1, HAS2, and HAS3) caused by UVB exposure and reduced UVB-induced collagen fiber degradation by inhibiting the expression of matrix metalloproteinase genes encoding MMP-1, MMP-2, and MMP-9. Meanwhile, topical treatments reduced cyclooxygenase-2 (COX-2) mRNA-level expression in photodamaged skin, leading to the inhibition of interleukin-1*β* (IL-1*β*) and interleukin-6 (IL-6) mRNA-level expression. Thus, ginseng phenolic acid-based preparations have potential value as topical treatments to protect skin against UVB-induced photoaging.

## 1. Introduction

In the human body, the skin is the largest organ. Skin provides a protective barrier against entry of toxins, pathogens, and environmental insults such as ultraviolet (UV) light [1, 2]. High-level UV irradiation, especially within the UVB wavelength range, is currently the most frequent cause of skin photodamage. From a clinical perspective, skin photodamage manifests as epidermal thickening accompanied by increased skin surface dryness, roughness, pigmentation irregularities, solar erythema, transepidermal water loss (TEWL), decreased elasticity, deep wrinkles, and other signs associated with premature aging [3–5]. Previous studies have demonstrated that visually apparent signs of UVB-induced skin damage result from irradiation-associated effects that trigger skin barrier dysfunction, skin dehydration, inflammation, and collagen degradation.

The article "Panax ginseng C. A. Meyer Phenolic Acid Extract Alleviates Ultraviolet B-Irradiation-Induced Photoaging in a Hairless Mouse Skin Photodamage Model" was published in 2021. Journal: Evid Based Complement Alternat Med.

When the body is exposed to UVB radiation, the skin barrier becomes compromised, resulting in decreased expression of filaggrin (FLG) protein and epidermal damage [6]. FLG, a key regulator of stratum corneum barrier function, undergoes cross-linking with transglutaminase-1 (TGM1) during formation of the cornified envelope that maintains skin moisture balance [7]. UVB-induced skin barrier damage leads to decreased skin moisture content due to reduced hyaluronic acid (HA) synthesis within the skin extracellular matrix (ECM) caused by decreased expression of hyaluronan synthases (HASs) present on the cytoplasmic side of skin cell plasma membranes [8]. Therefore, FLG, TGM1, and HASs are key players in the repair of skin barrier damage and maintenance of skin hydration function.

UVB radiation is known to stimulate cyclooxygenase-2 (COX-2) expression. COX-2, a proinflammatory mediator, stimulates the production of inflammatory cytokines tumor necrosis factor-*α* (TNF-*α*), interleukin-1*β* (IL-1*β*), and interleukin-6 (IL-6) [9, 10]. Entry of these cytokines into skin tissues leads to inflammatory damage and elevation of expression of various matrix metalloproteinases (MMPs) that degrade collagen fibers and accelerate skin photoaging [11–14]. MMPs are important enzymes with key roles in collagen-degradative processes that occur in the ECM, which is located within connective tissue [15, 16]. Researchers are currently devising strategies that reduce inflammation and MMPs activities toward preventing and treating skin photodamage after UVB exposure.

Due to their track record of safety and effectiveness, traditional Chinese medicinal extracts (TCM) have garnered increasing popularity for long-term use as daily topical skin-care treatments to prevent and alleviate skin photodamage. One such TCM, *Panax ginseng* C. A. Meyer has been used for many years as a skin conditioning treatment. Recently, compounds found in *Panax ginseng* extract have attracted attention due to their potentially beneficial biological activities [17]. In our previously reported work, we demonstrated that *Panax ginseng* phenolic acid extract (PG2) could inhibit melanogenesis via suppression of oxidative stress to lighten skin pigmentation in a B16 mouse melanoma cell-based skin hyperpigmentation model [18]. Meanwhile, other researchers have found that skin photoaging caused by UVB-irradiation exposure is closely linked to excessive production of reactive oxygen species (ROS) [19], suggesting that antioxidant compounds should be evaluated as treatments for skin photoaging. Due to the known antioxidant activities of phenolic acid compounds, here we evaluated PG2 and its main phenolic acid constituents to investigate their abilities to repair skin barrier damage, improve skin hydration, and alleviate MMPs- and inflammation-associated skin photoaging in a UVB-irradiated hairless mouse skin photodamage model.

The article "Panax ginseng C. A. Meyer Phenolic Acid Extract Alleviates Ultraviolet B-Irradiation-Induced Photoaging in a Hairless Mouse Skin Photodamage Model" was published in 2021. Journal: Evid Based Complement Alternat Med.

## 2. Materials and Methods

### 2.1. Chemicals and Reagents

Phenolic acid reference standards of ≥98% purity (caffeic acid, *p*-coumaric acid, protocatechuic acid, salicylic acid, and vanillic acid) were used in this study (Internet Aladdin Reagent Database Inc., Shanghai, China). Chloroform, ethyl acetate, and *n*-butanol (analytical grade) were obtained commercially (Beijing Chemical Works, Beijing, China). Acetonitrile and glacial acetic acid (HPLC grade) were purchased commercially (Merck, Darmstadt, Germany). The Magnetic Tissue/Cell/Blood Total RNA kit and FastKing cDNA Dispelling RT SuperMix kit used in this study were obtained commercially (TIANGEN, Beijing, China). The iTaq™ Universal SYBR® Green Supermix reagent was obtained commercially (Bio-Rad, CA, USA).

### 2.2. Preparation of Phenolic Acid-Containing *Panax ginseng* C. A. Meyer Extract and Its Major Phenolic Acid (PA) Constituents

PG2 was obtained using a previously reported method [18]. Briefly, after five-year-old ginseng plants were harvested, their roots were dried, cut into pieces, and then extracted in distilled water. Extracts were filtered to remove solids; then, filtrates were pooled then dried. Next, the remaining dried extracts were dissolved in distilled water; then, equal volumes of three solvents were added in succession to generate separate chloroform (first), ethyl acetate (second), and *n*-butanol (third) extracts. The ethyl acetate-derived extract described in this work, designated PG2, was characterized using two methods: high-performance liquid chromatography (HPLC) and liquid chromatography-mass spectrometry (LC-MS) [20, 21]. Ultimately, PG2 was shown to consist mainly of five phenolic acids that included caffeic acid, *p*-coumaric acid, protocatechuic acid, salicylic acid, and vanillic acid, with respective concentrations of 0.14 ± 0.01 g/100 g, 0.12 ± 0.01 g/100 g, 0.42 ± 0.02 g/100 g, 0.31 ± 0.02 g/100 g, and 6.85 ± 0.34 g/100 g. Next, these five acids were used to make standards by combining them in proportions based on their relative amounts (as they originally exist in PG2) to create PA.

The article "Panax ginseng C. A. Meyer Phenolic Acid Extract Alleviates Ultraviolet B-Irradiation-Induced Photoaging in a Hairless Mouse Skin Photodamage Model" was published in 2021. Journal: Evid Based Complement Alternat Med.

### 2.3. Source of Mice, Routine Animal Care, and Animal Experiments with PG and PA

Six-week-old female BALB/*c* hairless mice obtained commercially (Vital River Laboratory Animal Technology Co., Ltd., Beijing, China) were housed and cared for under 12-hour light/dark cycle conditions in an animal care facility. Guidelines of the National Institutes of Health Guide for the Care and Use of Laboratory Animals were followed for all experiments after approval of animal experimental methods was obtained from the Animal Ethics Committee of Changchun University of Chinese Medicine (Approval no. 20190119). Efforts were made to minimize the number of animals used in experiments and to minimize intensities of stimuli used.

Mice were assigned at random to five groups (*n* = 5). Experimental groups included the control (no UVB exposure, no treatment), UVB, UVB + Vehicle, UVB + PG2, and UVB + PA groups. Each mouse was weighed daily and its body weight was recorded. UVB skin exposure dose was measured to determine the minimal erythema dose (MED) for delivery of irradiation to mouse skin in the form of UVB radiation emitted by a UVB lamp (Hoefer Scientific Instruments, CA, USA). During the initial two days of experiments, skin on the back of each mice received a 1 MED (100 mJ/cm^2^) dose daily of UVB (except for the unirradiated control group). For the next two days, the daily UVB irradiation dose was delivered as before, but the dose was increased to 1.5 MED (150 mJ/cm^2^). Beginning on the 5th day, a daily dose of 200 mJ/cm^2^ was then applied until completion of experiments. According to the protocol regarding topical application of compounds to the skin of hairless mice [6], topical applications of PG2 (2 mg/cm^2^) and PA (2 mg/cm^2^) were applied daily after UVB exposure beginning on the 1st day for two weeks; meanwhile, topical application of 20% propylene glycol vehicle without PG2 or without PA was administered to the UVB + Vehicle group after UVB exposure for two weeks. Under isoflurane anesthesia, all mice in each group were examined to detect changes in skin morphology and skin surface physiological condition at completion of two-week treatments using a digital camera (EOS760D; Canon, Tokyo, Japan) and Cutometer^®^ Dual MPA 580 (Courage and Khazaka, Cologne, Germany). Then, all mice were sacrificed using CO_2_ asphyxiation for subsequent experiments [22].

### 2.4. Histological Evaluation

Dorsal skin specimens were harvested and then washed with PBS to remove any surface residues prior to histological examination. Next, skin specimens were fixed in 4% paraformaldehyde for 24 h and then were embedded in paraffin. Paraffin sections (3 *μ*m thick) were stained with hematoxylin and eosin (H&E) stain and Masson's trichrome stain followed by microscopic examination (TH4-200, Tokyo, Japan). For epidermal thickness determinations, thicknesses of skin tissues within each specimen were measured in *μ*m using a data analysis software package (Gen5, BioTek, VT, USA).

The article "Panax ginseng C. A. Meyer Phenolic Acid Extract Alleviates Ultraviolet B-Irradiation-Induced Photoaging in a Hairless Mouse Skin Photodamage Model" was published in 2021. Journal: Evid Based Complement Alternat Med.

### 2.5. Skin Surface Physiological Analysis

TEWL and water content of the stratum corneum were measured under standard environmental conditions (21–22°C and 50–55% humidity) using a Tewameter® TM 300 and a Corneometer® CM 825, respectively. Calculated TEWL and stratum corneum water content values were expressed in g/m^2^h and arbitrary units (AU), respectively, and then were compared among the five experimental groups.

### 2.6. Quantitative Real-Time PCR (qRT-PCR) Analysis

Dorsal skin total RNA was isolated using an Eppendorf epMotion M5073 nuclear purification workstation (Eppendorf, Hamburg, Germany) and a Magnetic Tissue/Cell/Blood Total RNA kit. After quantification of isolated total RNA was conducted via absorbance measurements at 260 nm, the RNA was reverse-transcribed using a FastKing cDNA Dispelling RT SuperMix kit. In order to investigate mRNA expression quantitatively, a CFX96 Touch Real-Time PCR Detection System (Bio-Rad, CA, USA) was used to conduct real-time PCR amplification of reactions containing iTaq™ Universal SYBR® Green Supermix. The 2^−ΔΔCt^ value method was used for data analysis, with results normalized to *β*-actin expression levels. The primer sequences are listed in Table 1.

### 2.7. Statistical Analysis

All data were expressed as mean ± SD. Statistical analysis was conducted using one-way analysis of variance (ANOVA), while multiple comparisons were conducted using Tukey's post hoc test using GraphPad Prism 7.0 (GraphPad Software, San Diego, CA, USA). *p* values < 0.05 were deemed statistically significant.

## 3. Results

### 3.1. Photoprotective Effects of PG2 and PA on Skin Photodamage Induced by UVB Exposure as Revealed by Morphological and Histological Examinations

Here, PG2 and PA restorative effects on UVB-induced skin photodamage were assessed *in vivo* by exposing skin of hairless mice to UVB irradiation and then treating the exposed skin with PG2, PA, or no treatment for two weeks. Throughout the experimental time period, different group mouse body weights were similar among the groups (Figure 1(a)). In the UVB-exposed group, dorsal skin signs of photodamage were apparent after irradiation, including increased dryness, roughness, and desquamation as compared to dorsal skin appearance of untreated, unirradiated (normal) mice. By contrast, topically applied PG2 and PA led to improvement of skin damage signs in UVB-irradiated mice. PG2, a natural phenolic acids source, thus appears to provide protect skin against photodamage, an effect that might be largely attributable to the activity of PA, its main phenolic acid constituents. Further support for this speculation lies in the fact that no overall differences in dorsal skin appearance were observed after two weeks of treatment with PG2 or PA (Figure 1(b)).

The article "Panax ginseng C. A. Meyer Phenolic Acid Extract Alleviates Ultraviolet B-Irradiation-Induced Photoaging in a Hairless Mouse Skin Photodamage Model" was published in 2021. Journal: Evid Based Complement Alternat Med.

In order to explore topical PG2 and PA treatment-associated suppression of epidermal thickening, we stained BALB/c hairless mouse dorsal skin sections from mice in each experiment group with H&E stain and then measured epidermal thickness in each skin specimen. Histological examination revealed greater epidermal thickness in UVB-exposed skin than in skin specimens of the control group. Intriguingly, as compared to the UVB + Vehicle group, PG2 and PA treatment groups exhibited more pronounced signs of recovery from UVB-induced pathological changes, with no significant differences in results found in the specimens of PG2 and PA groups (Figures 1(c) and 1(d)).

### 3.2. Restoration of TEWL and Stratum Corneum Water Content by Topical PG2 and PA Applications to UVB-Irradiated Dorsal Skin Areas of BALB/c Hairless Mice

In order to examine topical PG2 and PA treatment effects on skin photodamage, TEWL and stratum corneum water content were measured. After two weeks of UVB irradiation, TEWL increased and stratum corneum water content decreased. By contrast, topical PG2 and PA applications led to significant reductions of UVB-induced TEWL while improving water content of the stratum corneum. No significant differences among results obtained for PG2 and PA groups were found (Figures 2(a) and 2(b)).

### 3.3. Increased mRNA Expression of Genes Associated with Skin Barrier and Skin Hydration Functions in UVB-Exposed Skin of Hairless Mice after PG2 and PA Treatments

We examined mRNA-level expression of skin barrier-related genes encoding FLG and TGM1 and skin hydration-related genes encoding HASs to assess the effects of PG2 and PA on repair of skin barrier photodamage and impaired skin hydration after UVB exposure. The results revealed that mRNA-level expression of genes encoding FLG and TGM1 was significantly decreased in UVB-irradiated mouse skin tissues, while the expression levels of these mRNAs were significantly increased after skin was treated with PG2 and PA (Figures 3(a) and 3(b)). In addition, PG2 and PA treatments boosted mRNA-level expression of genes encoding HAS1, HAS2, and HAS3 that had decreased after UVB exposure, with the same effect observed in both PG2 and PA groups (Figures 3(c)–3(e)). Our results suggest that PG2 and PA can repair skin photodamage by restoring skin barrier function and improving skin hydration.

The article "Panax ginseng C. A. Meyer Phenolic Acid Extract Alleviates Ultraviolet B-Irradiation-Induced Photoaging in a Hairless Mouse Skin Photodamage Model" was published in 2021. Journal: Evid Based Complement Alternat Med.

### 3.4. Skin Collagen Fiber Density Was Restored in PG2- and PA-Treated UVB-Irradiated BALB/c Hairless Mouse Skin

After repeated exposure to UVB radiation, degradation of dermal collagen occurs that leads to reduced spatial density of collagen fibers [23]. In order to assess the effects of PG2 and PA treatments on collagen degradation induced by UVB exposure, BALB/c hairless mouse dorsal skin sections from all experimental groups were stained with Masson's trichrome stain. As shown in Figure 4, collagen fiber reductions and irregular collagen fiber distributions occurring after UVB exposure were restored to normal levels after topical PG2 and PA treatments. Thus, PG2 and PA treatments can prevent collagen degradation in mouse skin tissue after exposure to UVB radiation.

### 3.5. Downregulation of MMPs mRNA Expression in Skin of UVB-Irradiated Hairless Mice after PG2 and PA Treatments

After skin is exposed to UVB radiation, cytokine release triggers MMP expression [24]. Here, we measured mRNA levels reflecting expression of genes encoding MMP-1, MMP-2, and MMP-9 in dorsal skin tissues after the tissues were exposed to UVB radiation in order to investigate the effects of PG2 and PA on UVB-induced MMPs levels. In the UVB group, mRNA levels reflecting expression of genes encoding MMP-1, MMP-2, and MMP-9 significantly increased as compared with control group levels, with no significant differences observed among UVB and UVB + Vehicle groups. By contrast, topical skin treatment with PG2 or PA led to decreased mRNA-level expression of genes encoding these MMPs in dorsal skins as compared with corresponding levels for the UVB + Vehicle group, with no significant differences in results found among PG2 and PA groups (Figures 5(a)–5(c)). These results suggest that PG2 and PA protective effects may partially result from inhibition of MMPs release triggered by UVB exposure.

### 3.6. Decreased mRNA Expression of COX-2 and Proinflammatory Factor Genes (IL-1*β*, IL-6) in UVB-Exposed Skin of Hairless Mice after PG2 and PA Treatments

Results of several studies suggest that UVB irradiation of skin results in epidermal proliferation and elevated COX-2 expression [4]. Indeed, we observed that PG2 and PA treatments markedly inhibited COX-2 increases in UVB-induced skin tissues (Figure 6(a)). Furthermore, PG2 and PA treatments applied after UVB exposure led to markedly reduced IL-1*β* and IL-6 mRNA levels in skin, with no significant mRNA-level differences observed among PG2-and PA-treated groups (Figures 6(b) and 6(c)). Taken together, these results show reduced mRNA-level expression of genes encoding COX-2, IL-1*β*, and IL-6 in skin after treatment with PG2 and PA. Therefore, PG2 and PA may provide protection from inflammation occurring in UVB-irradiated skin by inhibiting production of these inflammatory mediators.

The article "Panax ginseng C. A. Meyer Phenolic Acid Extract Alleviates Ultraviolet B-Irradiation-Induced Photoaging in a Hairless Mouse Skin Photodamage Model" was published in 2021. Journal: Evid Based Complement Alternat Med.

## 4. Discussion

In our previous studies of PG2 effects on B16 mouse melanoma cells *in vitro*, PG2 was shown to possess antioxidant activity [18]. These results suggested that PG2 treatment might exert an antiphotoaging effect when administered *in vivo*. Due to the fact that PG2 isolated from ginseng contains natural phenolic acids, PG2 was evaluated using a UVB-induced photoaging hairless mouse model of skin damage. Intriguingly, both PG2 and its main phenolic acid constituents, PA, provided similar degrees of protection to prevent skin barrier damage, skin hydration impairment, collagen fiber degradation, and skin inflammation. These results indicated that phenolic acids present in PG2 may be largely responsible for observed PG2-protective effects against UVB-induced photodamage when applied to UVB-irradiated skin.

UVB radiation is known to greatly alter skin characteristics by triggering physiological changes of skin surface properties, histological features, and moisture loss [25,26]. Moreover, skin photodamage has been shown by some researchers to be linked to epidermal thickening that commonly occurs in UVB-irradiated skin [27,28]. By contrast, in PG2- or PA-treated mice, no apparent skin dryness and skin desquamation were observed, while epidermal thickness and TEWL values decreased and stratum corneum water content increased. Therefore, topical skin treatment with either PG2, or its main phenolic fraction PA, induced macroscopic repair of photodamaged skin resulting from UVB exposure.

Excessive UVB radiation can lead to skin barrier damage and skin dehydration by increasing TEWL and decreasing stratum corneum water content [29]. Therefore, we investigated the expression of genes encoding skin barrier- and skin hydration-related factors, such as FLG, TGM1, and HASs. Our studies have shown that PG2 and PA can improve skin barrier function and increase skin hydration to reduce skin photodamage by upregulating the expression of these factors.

Major photoaging characteristics of collagen fiber degradation and damage that occur in sunburned human skin have been shown to result from collagen extracellular matrix damage leading to reduced collagen and elastin levels [30,31], aligning with UVB group results in this work. Here, topical PG2 or PA treatments reversed decreases in collagen fiber number and density found in UVB-exposed skin to subsequently restore dermal collagen levels and skin structure. Therefore, topical administration of PG2 and PA treatments prevented skin photodamage by increasing dermal collagen density after skin exposure to UVB radiation.

The article "Panax ginseng C. A. Meyer Phenolic Acid Extract Alleviates Ultraviolet B-Irradiation-Induced Photoaging in a Hairless Mouse Skin Photodamage Model" was published in 2021. Journal: Evid Based Complement Alternat Med.

Histopathologically, collagen degradation resulting from elevated MMPs expression in UVB-irradiated skin is a key process that occurs during skin photoaging [32]. ECM-containing degradation targets of MMPs that have roles in the photoaging process include collagen, fibronectin, elastin, and proteoglycans [33]. In this study, UVB irradiation induced abnormally elevated levels of secreted MMP-1, MMP-2, and MMP-9, while PG2 and PA treatments of UVB-irradiated mice reversed upregulation of mRNA-level expression of MMPs-encoding genes. Collectively, these results align with our previous findings and suggest that PG2 and PA antioxidant and anti-inflammatory activities may account for their *in vivo* protective effects that act by reducing mRNA-level expression of genes encoding MMPs.

Exposure of skin to intense UVB irradiation has been shown to accelerate the production of proinflammatory cytokines (IL-1*β*, IL-6, and TNF-*α*) that trigger MMPs production. COX-2, a key enzyme involved in inflammation, is induced during inflammatory responses [4,34]. Meanwhile, IL-1*β* and IL-6 proinflammatory cytokines are integral participants in photoaging processes occurring within irradiated skin in the UVB-induced mice model such that UVB exposure appears to disrupt skin immune system function by increasing levels of proinflammatory cytokines [9,35,36]. In this study, treatment with PG2 or PA relieved UVB-induced immune system disruption and inflammation by reducing levels of COX-2, IL-1*β*, and IL-6 mRNAs, thus providing evidence to support the premise that PG2 and PA protect skin against photoaging by inhibiting these inflammatory mediators production.

## 5. Conclusions

Here, we demonstrated that PG2, a *Panax ginseng* phenolic acid extract, could protect skin of UVB-irradiated BALB/c hairless mice against photodamage. This effect was largely attributable to the effects of PA, the main phenolic acid constituents of PG2. This study highlights the potential value of ginseng phenolic acids for use as cosmetic additives toward the formulation of topical cosmeceuticals that can repair photodamaged skin.

## Figures and Tables

**Figure 1:** Topical applications of PG2 and PA improved skin health of UVB-photodamaged skin as assessed from morphological and histological observations. (a) Body weights during the experimental period. (b) Photographic images of dorsal skin in BALB/c hairless mice after two weeks. (c) H&E staining results after topical applications of PG2 and PA for two weeks. Scale bar: 100 *μ*m. (d) Quantitative analysis of epidermal thickness. Values are expressed as mean ± SD (*n* = 5). ^#^*p* < 0.05 versus the control group; ^*∗*^*p* < 0.05 versus the UVB + Vehicle group.

The article "Panax ginseng C. A. Meyer Phenolic Acid Extract Alleviates Ultraviolet B-Irradiation-Induced Photoaging in a Hairless Mouse Skin Photodamage Model" was published in 2021. Journal: Evid Based Complement Alternat Med.

**Figure 2:** Topical applications of PG2 and PA decreased TEWL values (a) and increased stratum corneum water content (b) in UVB-induced BALB/c hairless mice dorsal skin. Values are expressed as mean ± SD (*n* = 5). ^##^*p* < 0.01 and ^###^*p* < 0.001 versus the control group; ^*∗*^*p* < 0.05 versus the UVB + Vehicle group.

**Figure 3:** PG2 and PA treatments increased mRNA-level expression of genes encoding FLG, TGM1, HAS1, HAS2, and HAS3 in dorsal skin of UVB-irradiated hairless mice. mRNA levels of reflecting expression of genes encoding FLG (a), TGM1 (b), HAS1 (c), HAS2 (d), and HAS3 (e) were quantified using qRT-PCR after normalization of results to *β*-actin mRNA expression levels (internal control). Values are expressed as mean ± SD (*n* = 5). ^#^*p* < 0.05, ^##^*p* < 0.01, and ^###^*p* < 0.001 versus the control group; ^*∗*^*p* < 0.05 and ^*∗∗*^*p* < 0.01 versus the UVB + Vehicle group.

**Figure 4:** Topical applications of PG2 and PA blocked collagen degradation in UVB-irradiated mice skin. Collagen fibers were detected using Masson's trichrome staining method (*n* = 5). Scale bar: 100 *μ*m.

**Figure 5:** PG2 and PA treatments reduced mRNA-level expression of genes encoding MMP-1, MMP-2, and MMP-9 in dorsal skin of UVB-irradiated hairless mice. mRNA-level expression of genes encoding MMP-1 (a), MMP-2 (b), and MMP-9 (c) was quantified by qRT-PCR after normalization to *β*-actin mRNA expression levels (internal control). Values are expressed as mean ± SD (*n* = 5). ^##^*p* < 0.01 versus the control group; ^*∗*^*p* < 0.05 and ^*∗∗*^*p* < 0.01 versus the UVB + Vehicle group.

**Figure 6:** PG2 and PA treatments reduced mRNA-level expression of genes encoding COX-2, IL-1*β*, and IL-6 in dorsal skin of UVB-irradiated hairless mice. Levels of mRNA expressed by genes encoding COX-2 (a), IL-1*β* (b), and IL-6 (c) after normalization to *β*-actin mRNA expression levels (internal control). Values are expressed as mean ± SD (*n* = 5). ^#^*p* < 0.05, ^##^*p* < 0.01, and ^###^*p* < 0.001 versus the control group; ^*∗*^*p* < 0.05 and ^*∗∗*^*p* < 0.01 versus the UVB + Vehicle group.

**Table 1:** Primer sequences used for quantification of gene expression.

Gene	Sequence
MMP-1	Forward 5′-TTGCCCAGAGAAAAGCTTCAG-3′
	Reverse 5′-TAGCAGCCCAGAGAAGCAACA -3′

MMP-2	Forward 5′-CAGGGAATGAGTACTGGGTCTATT-3′
	Reverse 5′-ACTCCAGTTAAAGGCAGCATCTAC-3′

MMP-9	Forward 5′-AATCTCTTCTAGAGACTGGGAAGGAG-3′
	Reverse 5′-AGCTGATTGACTAAAGTAGCTGGA-3′

COX-2	Forward 5′-TGCTGTACAAGCAGTGGCAA-3′
	Reverse 5′-GCAGCCATTTCCTTCTCTCC-3′

IL-1*β*	Forward 5′-CAACCAACAAGTGATATTCTCCATG-3′
	Reverse 5′-AGATCCACACTCTCAGCTGCA-3′

IL-6	Forward 5′-GAGGATACCACTCCCAACAGACC-3′
	Reverse 5′-AAGTGCATCATCGTTGTTCATACA-3′

FLG	Forward 5′-ATGTCCGCTCTCCTGGAAAG-3′
	Reverse 5′-TGGATTCTTCAAGACTGCCTGTA-3′

TGM1	Forward 5′-TCTGGGCTCGTTGTTGTGG-3′
	Reverse 5′-AACCAGCATTCCCTCTCGGAT-3′

HAS1	Forward 5′-CACCATCTCAGCCTACCAAGA-3′
	Reverse 5′-ATCGGCGAAGACTTCTCGGA-3′

HAS2	Forward 5′-GAGCACCAAGGTTCTGCTTC-3′
	Reverse 5′-CTCTCCATACGGCGAGAGTC-3′

HAS3	Forward 5′-CCTGGAGCACCGTCGAATG-3′
	Reverse 5′-CCTTGAGGTTTGGAAAGGCAA-3′

*β*-Actin	Forward 5′-ATCACTATTGGCAACGAGCG-3′
	Reverse 5′-TCAGCAATGCCTGGGTACAT-3′

The article "Panax ginseng C. A. Meyer Phenolic Acid Extract Alleviates Ultraviolet B-Irradiation-Induced Photoaging in a Hairless Mouse Skin Photodamage Model" was published in 2021. Journal: Evid Based Complement Alternat Med.

## Data Availability

All data used to support the findings of this study are available from the corresponding author upon reasonable request.
